RETRACTED

# Effects of the Forecasting Methods, Precipitation Character, and Satellite Resolution on the Predictability of Short-Term Quantitative Precipitation Nowcasting (QPN) from a Geostationary Satellite

**DOI:** 10.1371/journal.pone.0140044

**Published:** 2015-10-08

**Authors:** Yu Liu, Du-Gang Xi, Zhao-Liang Li, Wei Ji

**Affiliations:** 1 Institute of Remote Sensing and Digital Earth, Chinese Academy of Sciences, Beijing, China; 2 Institute of Geographic Sciences and Natural Resources Research, Chinese Academy of Sciences, Beijing, China; 3 The PLA Information Engineering University, Zhengzhou, China; 4 Naval Institute of Hydrographic Surveying and Charting, Tianjin, China; 5 Key Laboratory of Agri-informatics, Ministry of Agriculture / Institute of Agricultural Resources and Regional Planning, Chinese Academy of Agricultural Sciences, Beijing, China; 6 ICube, UdS, CNRS, 300 boulevard Sebastien Brant, CS 10413, 67412, Illkirch, France; The Ohio State University, UNITED STATES

## Abstract

The prediction of the short-term quantitative precipitation nowcasting (QPN) from consecutive gestational satellite images has important implications for hydro-meteorological modeling and forecasting. However, the systematic analysis of the predictability of QPN is limited. The objective of this study is to evaluate effects of the forecasting model, precipitation character, and satellite resolution on the predictability of QPN usingimages of a Chinese geostationary meteorological satellite Fengyun-2F (FY-2F) which covered all intensive observation since its launch despite of only a total of approximately 10 days. In the first step, three methods were compared to evaluate the performance of the QPN methods: a pixel-based QPN using the maximum correlation method (PMC); the Horn-Schunck optical-flow scheme (PHS); and the Pyramid Lucas-Kanade Optical Flow method (PPLK), which is newly proposed here. Subsequently, the effect of the precipitation systems was indicated by 2338 imageries of 8 precipitation periods. Then, the resolution dependence was demonstrated by analyzing the QPN with six spatial resolutions (0.1atial, 0.3a, 0.4atial rand 0.6). The results show that the PPLK improves the predictability of QPN with better performance than the other comparison methods. The predictability of the QPN is significantly determined by the precipitation system, and a coarse spatial resolution of the satellite reduces the predictability of QPN.

## Introduction

The extrapolation-based short-term Quantitative Precipitation Nowcasting (QPN), which involves forecasting future precipitation in a notably short time (e.g., 0~2 hr) based on extracting information from current observations (e.g., radar and satellite imageries), is important for numerous hydro-meteorological applications [1, 2]. QPN can play a complementary role for Numerical Weather Prediction (NWP) models in quantitative precipitation forecasting [1] for capability of producing reliable nowcasting precipitation data, particularly for the analysis of a few hours [3–7].

RETRACTED

The predictability of precipitation study began in 1976 when the McGill Weather Radar Observatory started sending 1–6 hours of rainfall forecast to the local weather office [8]. Since then, various extrapolation-based algorithms have been proposed [9–12] and the predictability of QPN has been discussed to some extent [10–12, 13–17]. In contrast to numerous studies on the radar, much less effort has been devoted to geostationary satellite, although satellite-based QPN can provide data globally, particularly for regions lacking in situ observational systems such as rain gauge networks. In addition, the QPN method based on radar data always has challenge in applying in satellite because of demanding higher accuracy on tracking methods on sub-pixel level for small movement speed of clouds with coarser spatial resolution. On the other hand, smoother spatial characteristics of satellite products tend to make it harder to track cloud movement in the overlap region of two consecutive images for lack of obvious tracking signs compared to an equivalent terrestrial radar product.

Predictability of precipitation is a fundamental and intrinsic property of nonlinear systems stemming from complex dynamic and microphysical processes. Its prediction accuracy and computational time consumption depend on the particular forecasting model and the performance of the QPN methods. In addition, it is also closely related to the scanning scale of sensor. Thus, the understanding of the predictability should be made considering a specific method at a certain scale.

However, the precipitation forecast skill was always analyzed for only a single aspect such as the rainfall pattern, scale dependence, etc. [10–12, 18] Few studies were performed to systematically analyze the performance of different nowcasting models, although selecting a proper method is notably important to improve the predictability. It is of particular interest to determine the predictability of QPN from a comprehensive prospective. Therefore, the objective of this study was to analyze factors affecting the predictability of QPN systematically from forecasting model, precipitation system, and satellite resolution based on a new algorithm, pixel-based QPN using Pyramid Lucas-Kanade Optical Flow method (PPLK) proposed by the authors which was introduced in the following part.

RETRACTED

In this paper, section 2 describes the applied data sets and cases and section 3 presents the methodology. Section 4 reports the effects of the forecasting model, precipitation system, and satellite resolution on the predictability of QPN. Section 5 summarizes the work and outlines the conclusion.

## Data

Fengyun-2F (FY-2F) is the fourth operational geostationary meteorological satellite in China and was launched on 13 January 2012 in China. The FY-2F can scan typhoons, strong convection and other weather disasters with a high temporal resolution of 6–12 min/scan according to its observation task in the summer. This study collected all 6-min intensive observation data during 2013, which were composed of 2338 FY-2F precipitation estimation imageries of 8 periods with 0.01° spatial resolution, as shown in Table 1 (S1 Dataset). The precipitation estimation was made with a statistical regression model based on gauge rain and muti-channel infra-red light temperature data (10.3–11.3 μm, 11.5–12.5 μm, and 6.3–7.6 μm). There was significant intrinsic uncertainty in the precipitation estimation of FY-2F for the cloud-height-based methods as other geostationary satellite. Because of the high frequency and large spatial scale of FY-2F, the observations data (eg. radar, gauge and other satellite data) can hardly be match. Thus, this paper didn’t carry out the verification of FY-2F precipitation product.

**Table 1:** Information for the rainfall images of 8 periods in 2013 using Fengyun-2F (FY-2F), which include the time, length, spatial coverage, and main cloud types of the precipitation systems.

Rainfall event	Time (mmddhhmm) *	Length (hour)	Spatial coverage	The main cloud types **
T1	07170600–07181554	34.1	60°~160°E, 12°~50°N	Large-scale, enhanced Cumulonimbus, Altocumulus and Cumulus congestus
T2	07240400–07251154	31.9	60°~160°E, 25°~50°N	Small-scale Cumulonimbus,Cumulus Congestus
T3	08010412–08030354	47.8	60°~160°E, 10°~50°N	Large-scale Cumulonimbus, Altocumulus, and Altostratus
T4	08051200–08071154	48.0	60°~160°E, 5°~50°N	Small-scale and enhanced Cumulonimbus, Cumulus congestus
T5	08120400–08121148	8.0	60°~160°E, 10°~50°N	Large-scale, enhanced Cumulonimbus, Altostratus
T6	09200400–09200936	5.5	60°~160°E, 10°~50°N	Large-scale, enhanced Cumulonimbus, Altostratus
T7	09220900–09230230	12.8	60°~160°E, 10°~50°N	Medium-scale, dissipating Cumulonimbus, Congestus, and Cumulus congestus
T8	10050306–10071454	45.7	60°~160°E, 18°~50°N	Small-scale dissipating fast-moving Cumulonimbus, Cumulus congestus

* mmddhhmm: Month day hour minute.

** The scale definition in this study, such as large, medium and small scales, is not strictly based on meteorology. It is a relative concept that considers the spatial distribution of cloud on a geostationary satellite.

RETRACTED

The precipitation estimation data were provided by the NMSC (national satellite meteorological center of Chinese Meteorological Agency). It could be free downloaded from the web site of http://www.nsmc.cma.gov.cn/ with only a registered user name). They covered a rectangular region of different latitudes between 0°N~50eN. Considering the co-existence of several storms in a single imagery, these 2338 imageries covered almost all precipitation types that occurred in China. Fig 1 is the estimated precipitation of FY-2F at representative times for the 8 studied periods. The storms in the second (T2) and eighth periods (T8) were mainly composed of relatively small-scale, fast-moving, and more complicated variation clouds than the other 6 periods.

**Fig 1:** Estimated precipitation of Fengyun-2F (FY-2F) at representative times for the 8 periods studied. (a-h) are precipitation imageries of T1, T2… and T8 which are the same as in Table 1. Δt =4 hours, and the spatial resolution is 0.1°×0.1°.

Considering the smoother spatial characteristics of geostationary precipitation, this study used three typical ground-based radar rainfall events (1500–2100 UTC on 4 September 2013, 0900–1400 on 3 July 2010 and 1400–1720 on 7 June 2010) (S2 Dataset) to illustrate the effect of spatial resolution on QPN. They were provided by the Tsinghua University with spatial resolution 90 m and a frequency of 5min. The Radar covered a radius of 36km in the Tsinghua University, Beijing, China (116.32°E, and 40.01°N).

## Methodology

The predictability of QPN from the geostationary satellite can be analyzed from three perspectives: forecasting method, precipitation system, and satellite resolution.

A traditional QPN algorithm consists of a tracking and forecasting (extrapolation) process as suggested by Austin and Bellon [19]. Considering that the accuracy of precipitation advection was an important key limitation factor in QPN and the projection discontinuities was always produced during extrapolation, this study used a new algorithm: PPLK, which was proposed by the authors. The PPLK uses the pyramid Lucas-Kanade optical-flow method to improve the precipitation advection estimation and adds a new process called spatial interpolation to assign data to non-data rainy pixels. To further understand the effect of the QPN methods, this study compared the PPLK with two other typical methods: pixel-based QPN using the maximum correlation method (PMC) and the Horn-Schunck optical-flow method (PHS).

### 1. PMC

In general, the tracking method to detect cell patterns, whether radar- or satellite-data based, can be divided into two main techniques: pattern-oriented correlation techniques and overlapping techniques. PMC (S1 File) employs the former technique, a cross-correlation-based approach which is the most common technique for QPN (e.g., Tuttle and Foote [20]). It uses two successive estimated precipitation images to determine a displacement vector and identify the most matching locations based on dividing the entire domain of imagery into equally sized windows. On the first picture, digital image data of 3 × 3 pixels centered on the desired site are used as template data. On the second picture, taken one hour previously, image data of 15 × 15 pixels are used as search area. The correlation coefficient of estimated precipitation for the template area and the search area is calculated for each lag point to obtain a cross-correlation coefficient matrix, called a matching surface. The largest coefficient is adopted as the best-matched position at the pixel level. The forecasting process was identical to that of the PPLK, which was introduced in details in the following part.

RETRACTED

Considering the spatial resolution of precipitation estimation dataset of 0.1° (approximately 11.1 km×11.1 km at the equator, and approximately 5 km×5 km at 50°N in the latitudinal direction) and the temporal resolution of 6-min for the FY-2F, and a probable maximum wind speed of 150 m/s, the searching radius was set as 5 pixels for tracking clouds with moderate speeds.

### 2. PHS

The PHS (S1 File) is a more recent optical-flow-based method [21, 22] that tracks the clouds using a classical approach, the Horn-Schunck optical flow (HSOF) [23] to formulate the optical-flow constraint as a global variation problem to minimize the following cost function:

$$J=J_{0}+\alpha \times J_{HS}$$ (1)

where

$$J_{0}=\iint {\left[I_{t}+I_{x}u+I_{y}v\right]}^{2}dxdy$$ (2)

Ix, Iy, and It are the partial derivatives of x, y, and t for rainfall intensity, respectively. u and v are advection-field components in the x direction (west–east) and the y direction (north–south), respectively. JHS is a global constraint on the smoothness of the gradient of the optical flow field:

$$J_{HS}=\iint \left({\left|\nabla u\right|}^{2}+{\left|\nabla v\right|}^{2}\right)dxdy$$ (3)

Here, *α* is a tunable parameter that determines the weight of the smoothness term.

Because of the computationally expensive nature of the HSOF, this study divided the FY-2F imagery into several sub-windows. Thus, the window size of 50ry into several e smoothnboth the time consumption and the deformation of the cloud advection on the boundary of each window, for the QPN with larger sub-window size consumed more time which and smaller window size means more data for the deformation of the cloud advection on the boundary of each window. For example, the time consumption of QPN with lead time 120 min is 2.67 min and 24.51 min for the HSOF with sub-windows of 25×25 pixels and 50×50 pixels, respectively.

RETRACTED

### 3. PPLK

The PPLK (S3 File) uses the Lucas-Kanade Optical-Flow method [24] to locally resolve the aperture problem of the optical-flow constraint. Considering the limitation in tracking fast-moving objects with advection for more than one pixel because of the optical-flow constraint equation, this study used an image pyramid technique. The implementation of the PPLK was as follows:

#### (1) Pixel-based tracking

(a) Build pyramid: establish pyramid multi-resolution images of m+1 levels (level 0, 1…m) with FY-2F rainfall estimation images. Level m is the top of the pyramid. Level 0 is the bottom, which is also the original rainfall estimation image. In this study, 4 levels of pyramid images with spatial resolution of 0.1°, 0.2°, 0.3°and 0.4°from the bottom to the top were used. Their box sizes started at the full domain. (b) Estimate the derivative of a rainy pixel (k, l) with respect to the u_m_(k, l) in the x direction (west–east) and v_m_(k, l) in the y direction (north–south) for the top of the pyramid (level m) using LKOF with a Gaussian kernel before processing. (c) Assume the level m–1, m–2…0 is level i, and estimate the LKOF of pixel (k, l) at level i.

$$u_{i}(k,l)=u_{i}^{*}(k,l)+u_{i}^{\prime }(k,l)$$ (4)

$$v_{i}(k,l)=v_{i}^{*}(k,l)+v_{i}^{\prime }(k,l)$$ (5)

where $u_{i}^{*}(k,l)$ and $v_{i}^{*}(k,l)$ are the compensation optical flows of pixel (k, l) at level i. They are twice the compensation LKOF estimated at level i+1 using the bilinear interpolation method. $u_{i}^{\prime }(k,l)$ and $v_{i}^{\prime }(k,l)$ are the standard LKOFs of the compensated image of level i+1; repeat this step until finishing the estimation of the optical flow field for all pixels at level 0 (original image).

#### (2) Rainfall extrapolation

(a) Project the cloud forward and backward using the linear extrapolation method and the precipitation advection obtained in section 2.1 on the pixel level. In a forward scheme we start at purple pixels (t) and advect them downstream up to purple pixels (t+1). Whereas in a backward scheme, we move upstream and determine the origin purple pixels (t) that would end up at yellow grid points pixels (t–1). (b) Estimate precipitation evolution on assumption that rainfall rate varied linearly which can be calculated based on the observed and the backward forecasted precipitation at time t according to step (a). (c) Forecast rainfall intensity at time t+1 pixel-by-pixel considering the precipitation advection and evolution based on step (a) and step (b). It can be described as below:

$$P_{t+n\Delta t}(x_{t+n\Delta t},y_{t+n\Delta t})=\text{max}\left\{\text{min}\left[P_{t}(x_{t},y_{t})+n\Delta P,Threshold_{\text{max}}\right];Threshold_{\text{min}}\right\}\;$$ (6)

$$\left(x_{t+n\Delta t},y_{t+n\Delta t})=(x_{t},y_{t})+n\Delta (x_{t},y_{t}\right)$$ (7)

Where *P*_*t*+*n*Δ*t*_ is the predicted rain rate at *t*+*n*Δ*t*. (*x*_*t*+*n*Δ*t*,_ *y*_*t*+*n*Δ*t*_) is the predicted location of pixel (*x*_*t*_,*y*_*t*_). The *Threshold*_max_ and *Threshold*_min_ are the maximum and minimum possible rain rate of 50 mm/h and 0 mm/h.

RETRACTED

#### (3) Spatial interpolation

(a) Identify pixels in the extrapolation image that are neighboring in the previous image and determine whether the non-data pixels are located in the square. (b) Estimate the value of the identified pixels using inverse distance method assuming that the topological relationships of the cloud pixels do not change in consecutive images. (c) Repeat steps (a-b) until all pixels surrounded by four neighboring pixels are found.

### 4. Parameters and Analysis

The parameters of the PPLK are grouped into two categories:(a) Cloud advection estimation parameters: 4 pyramid levels; 5×5 searching windows; the matrices of the filter function in the extension process of the pyramid are (0.25 –alpha / 2, 0.25, alpha, 0.25, 0.25—alpha / 2), where alpha is 0.4. (b) Precipitation extrapolation parameter: the search radius of the spatial interpolation for the forecast image was set as “lead time × 3 / forecasting step + 6”.

The effect of the precipitation system is indicated by the storms of these 8 periods, which involve various cloud types and complex rapidly developing characters on both small and large scales, as shown in Fig 1 and Table 1.

To analyze the effect of the spatial resolution, this study resampled satellite precipitation estimation data from the native resolution (0.1°) to five spatial resolutions (0.2°, 0.3°, 0.4°, 0.5°and 0.6°) and compared it to the QPN of radar.

In addition, to further indicate the performance of PMC, PHS and PPLK, this study compared them with other methods in previous studies (e.g., Zahraei et al. 2013), although different cases were used. Because numerous images were used and there were several storms in a single imagery, the comparison was reasonable.

The predictability of the QPN from the satellite was demonstrated using six indices: relative bias (Bias), coefficient of correlation (Corr), normalized mean square error (NMSE), probability of detection (POD), false-alarm rate (FAR), and critical success index (CSI). The first two indices quantitatively measure the consistency between forecasting and observation. The POD, FAR, and CSI demonstrate the skill of predicting the occurrence of precipitation above a predefined threshold. For example, the POD shows the ability of the QPN algorithm to predict rainy/non-rainy pixels. The FAR indicates instances where the storm is predicted but there is no storm. The CSI shows how well the predicted storm corresponds to the observed storm. These indices are defined as:

$$Bias=\frac{\sum_{i=1}^{N}\overset{⌢}{P}(i)-\sum_{i=1}^{N}P(i)}{\sum_{i=1}^{N}P(i)}\times 100\text{\%}$$ (8)

$$Corr=\frac{\sum_{i=1}^{N}\left(P(i)\text{-}\bar{P}\right)\times \sum_{i=1}^{N}\left(\overset{⌢}{P}(i)\text{-}\overset{⌢}{\bar{P}}\right)}{\sqrt{\sum_{i=1}^{N}{\left(P(i)\text{-}\bar{P}\right)}^{2}\times \sum_{i=1}^{N}{\left(\overset{⌢}{P}(i)\text{-}\overset{⌢}{\bar{P}}\right)}^{2}}}$$ (9)

$$NMSE=\sqrt{\frac{\sum_{i=1}^{N}|\overset{⌢}{P}(i)\text{-}{P(i)|}^{2}}{N}}$$ (10)

$$POD=\frac{hits}{hits+misses}$$ (11)

$$FAR=\frac{falsealarms}{hits+falsealarms}$$ (12)

$$CSI=\frac{hits}{hits+misses+falsealarms}$$ (13)

where $\overset{⌢}{P}(i)$ and *P*(*i*) are the forecast and observed rainfall intensities of pixel *i*, respectively. *N* is the number of pixels in the prediction domain. $\overset{⌢}{\bar{P}}$ and $\bar{P}$ are the average forecast and observed precipitation, respectively. *hits*, *misses*, and *falsealarms* are the number of hits, failures, and false alarms, respectively. The Bias, NMSE and FAR of an ideal QPN algorithm should be 0, whereas the Corr, POD and CSI should be 1.

RETRACTED

## Results

### 1. Effects of the forecasting methods

Table 2 shows the comparisons of PPLK vs. PMC and PHS. The optical-flow-based QPN of both PPLK and PHS outperformed the PMC method with significant improvement in the predictability of QPN in terms of 6 measures over the 30–120 min lead time. For example, the average Bias of the QPN using MCM, PHS and PPLK was 89.96PHS an%, 14.82S an% and 8.75and P%, respectively, for 30 hours of lead time. The NMSE was 2.94 NMSE mm/h, 1.43 NMSE mm/h and 1.18.ely,Lmm/h, respectively. The other four measures (Corr, POD, FAR and CSI) over the QPN with 60–120 min lead time have similar variations.

**Table 2:** Average measures of PPLK, PMC, PHS and other short-term quantitative precipitation nowcasting (QPN) methods with 30 min, 60 min, 90 min and 120 min lead time.

Lead time (min)	Method*	Bias (%)	Corr	NMSE(mm/h)	POD	FAR	CSI
30	PMC	89.96mm/h)	0.696mm/h	2.946mm/h	0.986mm/h	0.576mm/h	0.426mm/h
	PHS	14.82mm/h	0.812mm/h	1.432mm/h	0.892mm/h	0.372mm/h	0.592mm/h
	PPLK	8.752mm/h	0.822mm/h	1.182mm/h	0.872mm/h	0.372mm/h	0.582mm/h
	PERCAST-GD				0.54~0.68	0.37~0.49	0.32~0.42
	PERCAST				0.50~0.62	0.44~0.53	0.36~0.25
	WDSS-II				0.58~0.46	0.45~0.55	0.19~0.32
	PER				0.41~0.51	0.49~0.58	0.16~0.22
60	PMC	180.55I122.24	0.5624I06	5.2324I43	0.9724I09	0.7724I1	0.3724I4
	PHS	28.184I9.08	0.6984I08	2.1584I0	0.7784I07	0.4484I07	0.4884I07
	PPLK	12.884I.72	0.7084I08	1.7284I8	0.7584I07	0.4384I07	0.4884I07
	PERCAST-GD				0.44~0.60	0.43~0.52	0.20~0.32
	PERCAST				0.39~0.52	0.52~0.60	0.16~0.25
	WDSS~II				0.38~0.47	0.54~0.62	0.14~0.20
	PER				0.30~0.36	0.60~0.68	0.08~0.12
90	PMC	259.24T195.43	0.4743T07	7.2543T46	0.9643T13	0.7643T12	0.2443T04
	PHS	51.223T8.61	0.5923T09	2.9423T40	0.7023T11	0.5223T09	0.4223T7
	PPLK	17.553T3.23	0.6353T9	2.1653T03	0.6753T09	0.5153T08	0.4153T7
120	PMC	323.59T232.51	0.4151.08	8.8951.08	0.9551.08	0.8051.08	0.2051.08
	PHS	81.841.08D1	0.5041.08	3.8041.0	0.6541.08	0.5941.08	0.3341.08
	PPLK	25.831.08D6	0.5131.08	2.5931.08	0.6131.08	0.5731.08	0.3431.08

*PPLK: Pixel-based QPN using the Pyramid Lucas-Kanade Optical-Flow method; MCM: Pixel-based QPN using the maximum correlation method; PHS: Pixel-based QPN using Horn-Schunck optical-flow method; PERCAST: PERsiann (Precipitation Estimation from Remotely Sensed Information using Artificial Neural Networks) - -ForeCAST; PERCAST-GD: PERsiann-ForeCAST considering the storm Growth and Decay (GD) whose area increases or decreases compared to previous moments; WDSS: Warning Decision Support System; PER: PERsistence. The PMC, PHS and PPLK were compared based on 2338 images of 8 periods of FY-2F in this paper. The PERCAST-GD, PERCAST, WDSS~II and PER was compared by Zahraei et al. [6] based on four storms from GOES-IR data over a rectangular region in 80–115°W and 32–45°N.

RETRACTED

Compared with the PHS, the PPLK performed better with obvious improvement in Bias and NMSE and slight improvement in Corr, POD, FAR and CSI.

The comparison with other methods from previous studies by Zahraei et al. [6] also shows that the PPLK method improved the predictability of the QPN. The accuracy of the 120-min QPN using PPLK was comparable to that of 30 min lead time using other methods considering the numerous images that were used and the co-existence of several storms in a single imagery. For example, the POD, FAR and CSI of the PPLK were 0.61esing other methodsm 0.34±0.07, respectively, for the 120-min QPN, whereas those of the PERCAST-GD (Precipitation Estimation from Remotely Sensed Information using Artificial Neural Networks considering storm-ForeCAST-Growth and Decay), which was the best of the four compared methods in Zahraei et al. [6], were 0.54~0.68, 0.37~0.49 and 0.32~0.42 for the QPN with 30 min lead time.

### 2. Effects of the precipitation character

Table 3 shows 6 average measures over 8 periods of QPN with 30 min, 60 min, 90 min, and 120 min lead time. Fig 2 shows the Corr and CSI of 2338 images. The measures significantly fluctuated, and the rainfall system significantly affected the predictability of the QPN. For example, using the PPLK, the average Bias, Corr, NMSE, POD, FAR and CSI of the 30 min QPN were 8.75in QP%, 0.82in QP, 1.18in 54 mm/h, 0.87, 54, 0.37, 54 and 0.58 54 wereR and CSI they were 12.88 54%, 0.788 5, 1.728 54mm/h, 0.758 54, 0.438 54, 0.488 54 for the 60 min lead time, respectively, and 25.83ective%, 0.5183ec, 2.5983ectimm/h, 0.61, ec, 0.57, ect, and 0.34tive7 for the 120 min lead time, respectively.

RETRACTED

**Table 3:** Average 6 measures of QPN with 30 min, 60 min, 90 min and 120 min lead time for 8 periods using the PPLK: coefficient of correlation (Corr), normalized mean square error (NMSE), probability of detection (POD), false-alarm rate (FAR), and critical success index (CSI).

Lead time (min)	Rainfall Event	Bias (%)	Corr	NMSE (mm/h)	POD	FAR	CSI
30	T1	10.82)%)ei	0.822)%)e	1.412)%)e	0.892)%)e	0.372)%)e	0.592)%)e
	T2	12.16)%)ei	0.716)%)e	0.466)%)	0.796)%)e	0.4460.06	0.4860.06
	T3	6.2460.06	0.8560.06	1.6660.06	0.9660.0	0.3360.06	0.6260.06
	T4	7.8560.0	0.8460.06	1.4460.	0.9460.0	0.3660.06	0.6660.0
	T5	7.6860.06	0.8660.06	1.9760.06	0.9160.06	0.3560.06	0.6260.06
	T6	3.8760.06	0.9760.0	1.7260.0	0.9360.06	0.2660.06	0.7660.0
	T7	8.8560.06	0.8560.06	1.4760.06	0.9160.06	0.3460.06	0.6260.06
	T8	9.1360.06	0.8260.06	0.5260.0	0.8560.06	0.3960.06	0.5560.06
	Average	8.75age06	0.82age06	1.18age06	0.87age06	0.37age06	0.58age06
60	T1	15.55ge06i	0.755ge0	2.045ge06	0.775ge06	0.435ge06	0.485ge06
	T2	18.53ge06iz	0.543ge06	0.653ge06	0.633ge06	0.553ge06	0.353ge06
	T3	9.353ge06	0.733ge06	2.493ge06	0.773ge06	0.393ge06	0.523ge06
	T4	11.32ge06i	0.722ge06	2.062ge06	0.772ge06	0.412ge06	0.512ge0
	T5	11.52ge06	0.742ge06	2.912ge06	0.79±0.03	0.49±0.0	0.52±0.03
	T6	5.27±0.03	0.81±0.03	2.52±0.0	0.83±0.03	0.33±0.0	0.61±0.03
	T7	12.430.03	0.7630.03	2.0330.03	0.8230.03	0.3830.03	0.5430.03
	T8	13.490.0	0.7490.0	0.7190.03	0.7390.03	0.4590.03	0.4690.03
	Average	12.88ge03i	0.788ge0	1.728ge0	0.75±0.07	0.43±0.07	0.48±0.07
90	T1	21.590.07i	0.6590.0	2.5690.07	0.6990.07	0.5190.07	0.4190.0
	T2	28.880.07i	0.4380.07	0.8280.07	0.5380.07	0.6480.07	0.2780.07
	T3	12.740.07i	0.6340.07	3.1740.07	0.6940.07	0.4740.07	0.4340.07
	T4	14.660.07i	0.6260.07	2.6±0.38	0.690.387	0.490.387	0.420.387
	T5	15.60.387	0.650.387	3.750.3	0.710.387	0.470.387	0.430.387
	T6	5.810.387	0.730.387	3.150.387	0.770.387	0.360.387	0.540.387
	T7	16.66.387i	0.696.387	2.466.387	0.776.387	0.446.387	0.486.387
	T8	16.61.387iz	0.661.38	0.851.387	0.651.387	0.511.387	0.381.387
	Average	17.55ge87iz	0.655ge8	2.165ge87	0.675ge87	0.515ge87	0.415ge8
120	T1	31.63ge87iz	0.513ge87	3.083ge87	0.643ge87	0.583ge87	0.343ge87
	T2	45343ge8	0.333ge87	0.983ge87	0.463ge8	0.723ge87	0.213ge87
	T3	19.11ge839	0.541ge83	3.811ge83	0.631ge83	0.541ge83	0.361ge83
	T4	20.91ge83	0.531ge83	3.131ge8	0.631ge83	0.551ge83	0.361ge83
	T5	22.06ge839z	0.566ge83	4.476ge83	0.656ge83	0.546ge83	0.376ge83
	T6	7.376ge83	0.656ge83	3.776ge83	0.716ge83	0.436ge83	0.466ge83
	T7	23.58±3.39	0.628±3.3	2.888±3.3	0.738±3.3	0.498±3.3	0.438±3.3
	T8	23.75±3.39z	0.525±3.3	1.525±	0.595±3.3	0.585±3.3	0.325±3.3
	Average	25.83ge.39z	0.513ge.	2.593ge.3	0.613ge.	0.573ge.3	0.343ge.3

RETRACTED

**Fig 2:** Coefficient of correlation (Corr) and critical success index (CSI) of QPN using Pyramid Lucas-Kanade Optical Flow method (PPLK) vs. 30 min, 60 min, 90 min and 120 min lead time. for 2338 images of 8 periods using Pixel-based.

For the rainfall events, the PPLK had a similar relatively good performance except for T2 and T8, which were composed of relatively small-scale, fast-moving Cumulonimbus and Cumulus Congestus and involved complicated development processes such as the new birth, dispersion and merging of cloud patches, as shown in Fig 1. The PPLK performed worse during T2 and T8 because the high spatiotemporal variability of the precipitation complicated the present study of QPN, where the cloud-tracking-based QPN methods treat a cloud patch as robust and assume that the relative positions of the cloud pixels do not change. However, it was observed that the birth, dispersion and merging of cloud patches widely occurred.

### 3. Effects of the satellite resolution

Fig 3 shows the average Corr and CSI of all events for 0–120 min predictions vs. the spatial resolution (0.1t, 0.2t, 0.3t, 0.4tial reand 0.6). Fig 4 is similar to Fig 3 but for 3 radar events for 0–60 min predictions vs. spatial resolution (90m, 180m, 270m, and 360m). The results show that the CSI and Corr of QPN decreases with coarser spatial resolutions, except for the spatial resolution of 0.1–0.2t, and that the Corr slightly increased with coarser spatial resolution.

**Fig 3:** Average Corr and CSI of all 8 events for 0–120 min predictions vs. different spatial resolutions of FY-2F using PPLK.

**Fig 4:** Average Corr and CSI of 3 events for 0–60 min predictions vs. different spatial resolutions of radar using PPLK.

The variation of QPN with different satellite resolutions is different from that of radar in Fig 4 in which Corr and CSI increases firstly then decreases with decreasing spatial resolutions, which means that QPN with radar medium spatial resolutions has better prediction skill which also could be found in other studies (Zahraei et al., 2012).

RETRACTED

The inconsistency of QPN for different spatial resolutions and between satellite and radar occurs because coarser resolutions can improve the QPN performance by reducing the image noise and decrease the accuracy of QPN by failing to track and forecast some small and metro-scale clouds, which spread over a few or a dozen pixels.

## Summary and Conclusions

In this study, the factors affecting the predictability of QPN ware analyzed using different QPN methods, precipitation characters and spatial resolution. The results show that:

1. The optical-flow-based QPN methods, i.e., PPLK and PHS, outperformed the PMC with significantly improved accuracy for 6 measures. Compared with the PHS, the PPLK performs better with obvious improvement in Bias and NMSE and slight improvement in Corr, POD, FAR and CSI. The PPLK with a 120-min lead time is comparable to the 30-min QPN of the other methods, although different cases and scans were used.
2. The coarser spatial resolution of the geostationary satellite generally reduces the predictability of QPN despite a slight improvement in Corr when the spatial resolution increases from 0.1°to 0.2°.
3. The rainfall system significantly affects the predictability of QPN, where the measure indices significantly fluctuate, and the QPN methods have limitations in predicting precipitation with high spatiotemporal variations.

## Supporting Information

S1 Dataset Estimated precipitation data of Fengyun-2F (FY-2F) of 8 periods in 2013 with an interval of 6-min. (RAR)

S2 Dataset Estimated precipitation data for three typical ground-based radar rainfall events with spatial resolution 90 m and a frequency of 5 min. (RAR)

S1 File The code and sample of the maximum correlation method (PMC) method. (RAR)

S2 File The code and sample of the Horn-Schunck optical-flow method (PHS). (RAR)

S3 File The code and sample of the Pyramid Lucas-Kanade Optical Flow method (PPLK). (RAR)

## References

[1] GangulyAR, BrasRL. Distributed quantitative precipitation forecasting using information from radar and numerical weather prediction models. Journal of Hydrometeorology, 2003; 4: 1168–1180. doi: 10.1175/1525-7541(2003)004<1168:DQPFUI>2.0.CO;2

[2] AfsharA, ZahraeiA, MariñoM. Large-scale nonlinear conjunctive use optimization problem: decomposition algorithm. Journal of Water Resources Planning and Management, 2010; 136: 59–71. doi: 10.1061/(ASCE)0733-9496(2010)136:1(59)

[3] LiangQ, FengY, DengW, HuS, HuangY, ZengQ, et al A composite approach of radar echo extrapolation based on TREC vectors in combination with model-predicted winds. Advances in Atmospheric Sciences, 2010; 27: 1119–1130. doi: 10.1007/s00376-009-9093-4

RETRACTED

[4] LiguoriS, Rico-RamirezMA, SchellartANA, SaulAJ. Using probabilistic radar rainfall nowcasts and NWP forecasts for flow prediction in urban catchments. Atmospheric Research, 2012;103: 80–95.

[5] SokolZ, PesiceP. Nowcasting of precipitation—advection statistical forecast model (SAM) for the Czech Republic. Atmospheric Research, 2012;103: 70–79.

[6] ZahraeiA, HsuK, SorooshianS, GourleyJJ, HongY, BehrangiA. Short-term quantitative precipitation forecasting using an object-based approach. Journal of Hydrology, 2013; 483:1–15

[7] ZahraeiA, HsuK, SorooshianS, GourleyJJ, HongY, LakshmananV, et al Short-term quantitative precipitation forecasting: a Lagrangian pixel based approach. Atmospheric Research, 2012;?: 418–434

[8] BellonA, AustinG L. The evaluation of two years of real-time operation of a short term precipitation forecasting procedure (SHARP). Journal of Applied Meteorology, 1978; 17:1778–1787. doi: 10.1175/1520-0450(1978)017<1778:TEOTYO>2.0.CO;2

[9] DixonM, WienerG. TITAN: thunderstorm identification, tracking, analysis and nowcasting–a radar-based methodology. Journal of Atmospheric and Oceanic Technology, 1993; 10:785–797. doi: 10.1175/1520-0426(1993)010<0785:TTITAA>2.0.CO;2

[10] GermannU, ZawadzkiI. Scale-dependence of the predictability of precipitation from continental radar images. Part I: description of the methodology. Monthly Weather Review. 2002; 130: 2859–2873. doi: 10.1175/1520-0493(2002)130<2859:SDOTPO>2.0.CO;2

[11] GermannU, ZawadzkiI. Scale-dependence of the predictability of precipitation from continental radar images. Part II: probability forecasts. Journal of Applied Meteorology. 2004; 43: 74–89. doi: 10.1175/1520-0450(2004)043<0074:SDOTPO>2.0.CO;2

[12] GermannU, ZawadzkiI, TurnerB. Predictability of precipitation from continental radar images. Part IV: limits to prediction. Journal of the Atmospheric Sciences, 2006; 63: 2092–2108. doi: 10.1175/JAS3735.1

[13] BellonA, LeeG, ZawadskiI. Error statistics of VPR corrections in stratiform precipitation. Journal of Applied Meteorology. 2005; 44: 998–1015. doi: 10.1175/JAM2253.1

[14] LiL, SchmidW, JossJ. Nowcasting of Motion and Growth of Precipitation with Radar over a Complex Orography. Journal of Applied Meteorology, 1995;34: 1286–1300. doi: 10.1175/1520-0450(1995)034<1286:NOMAGO>2.0.CO;2

[15] MecklenburgS, JossJ, SchmidW. Improving the nowcasting of precipitation in an Alpine region with an enhanced radar echo tracking algorithm. Journal of Hydrology, 2000; 239: 46–68. doi: 10.1016/S0022-1694(00)00352-8

[16] SeedAW. A dynamic and spatial scaling approach to advection forecasting. Journal of Applied Meteorology. 2003; 42: 381–388. doi: 10.1175/1520-0450(2003)042<0381:ADASSA>2.0.CO;2

RETRACTED

[17] TurnerB, ZawadzkiI, GermannU. Predictability of precipitation from continental radar images. Part III: Operational nowcasting implementation (MAPLE). Journal of Applied Meteorology, 2004; 43: 231–248. doi: 10.1175/1520-0450(2004)043<0231:POPFCR>2.0.CO;2

[18] LiuY, XiDG, LiZL, ShiCX. Analysis and Application of the Relationship between Cumulonimbus (Cb) Cloud Features and Precipitation Based on FY-2C Image. Atmosphere, 2014; 5: 211–229. doi: 10.3390/atmos5020211#sthash.5QLNqp0T.dpuf

[19] AustinGL, BellonA. The use of digital weather records for short term precipitation forecasting. Quarterly Journal of the Royal Meteorological Society, 1974; 100: 658–664. doi: 10.1002/qj.49710042612

[20] TuttleJD, FooteGB. Determination of the boundary layer airflow from a single Doppler radar. Journal of Atmospheric and Oceanic Technology, 1990; 7:218–232. doi: 10.1175/1520-0426(1990)007<0218:DOTBLA>2.0.CO;2

[21] CheungP, YeungHY. Application of optical-flow technique to significant convection nowcast for terminal areas in Hong Kong. The 3rd WMO International Symposium on Nowcasting and Very Short-Range Forecasting (WSN12), 2012; pp. 6–10

[22] HanL, WangHQ, LinYJ. Application of Optical Flow Method to Nowcasting Convective Weather. Acta Scientiarum Naturalium Universitatis Pekinensis, 2008;44:751–755 (in Chinese with English abstract)

[23] HornBK, SchunckBG. Determining optical flow. Artificial Intelligence, 1981; 17: 185–203. doi: 10.1117/12.965761

[24] LucasBD, KanadeT. An iterative image registration technique with an application to stereo vision. Proceedings of Seventh International Joint Conference on Artificial Intelligence, 1981; 81:674–679

